RETRACTED

# Chondro-protective effects of polydatin in osteoarthritis through its effect on restoring dysregulated autophagy via modulating MAPK, and PI3K/Akt signaling pathways

**DOI:** 10.1038/s41598-019-50471-y

**Published:** 2019-09-25

**Authors:** Zhengyuan Wu, Zhiwei Luan, Xiaohan Zhang, Kai Zou, Shiting Ma, Zhenyi Yang, Wenyu Feng, Mingwei He, Linhua Jiang, Jia Li, Jun Yao

**Affiliations:** 1 Department of Orthopaedics Trauma and Hand Surgery, The First Affiliated Hospital of Guangxi Medical University, Nanning, 530021 China; 2 Department of Bone and Joint Surgery, The First Affiliated Hospital of Guangxi Medical University, Nanning, 530021 China; 3 Departments of Pathology, The First Affliated Hospital of Guangxi Medical University, Nanning, 530021 China; 4 Guangxi Collaborative Innovation Center for Biomedicine, Life Sciences Institute, Guangxi Medical University, Nanning, 530021 China

**Keywords:** Drug development, Cartilage, Osteoarthritis

## Abstract

Osteoarthritis (OA) is a degenerative disease of the cartilage that is prevalent in the middle-aged and elderly demography. Polydatin (PD), a natural resveratrol glucoside, has shown significant anti-inflammatory and anti-arthritic potential in previous studies. This study was designed to evaluate the therapeutic properties of PD *in vitro* and *in vivo*, and elucidate their underlying mechanisms. The expression levels of all relevant factors were evaluated by qRT-PCR, western blotting, and immunohistochemistry (IHC) where suitable. Reactive oxygen species (ROS) and apoptosis were analyzed using the suitable probes and flow cytometry. The histological evidence of cartilage was assessed in rat models, moreover, the several serum cytokines levels and autophagy levels were evaluated. The result showed PD displayed significant chondro-protective effects, inferred in terms of reduced inflammation and cartilage degradation, apoptosis inhibition, and lower ROS production. The protective effects were attenuated by the autophagy inhibitor 3-MA, indicating a mediating role of autophagy in PD action. Mechanistically, PD exerted its effects by inhibiting the MAPK and PI3K/Akt signaling pathways which led to the down-regulation of mTOR. In conclusion, PD protects against cartilage degeneration by activating the autophagy flux in the chondrocytes via the MAPK and PI3K/Akt signaling pathways.

## Introduction

Osteoarthritis (OA) is a disease in which joints undergo chronic degeneration, particularly in older adults, with upwards of 15% of the world being affected by OA^1,2^. OA is primarily associated with breakdown of the articular cartilage owing to extracellular matrix (ECM) loss and substantial fibrotic development, resulting in eventual total cartilage loss^3^. While some medications can reduce OA symptoms via affecting the subchondral bone and synovium, there is currently a lack of effective therapies owing to its complex pathology. In addition, the drugs often cause severe complications including gastrointestinal bleeding and cardiovascular diseases^4–6^. Individuals with advanced OA require surgery to replace joints with prosthetic alternative and may require arthroscopic surgery^7,8^. Plant-derived agents have increasingly gained attention as a viable therapeutic alternative due to their minimum side effects and low costs^9^.

RETRACTED

Polydatin (PD) or 3,4′0.5-trihydroxystilbene-3-β-D-glucoside is a natural compound extracted from the roots of *Polygonum cuspidatum*, and has documented anti-inflammatory, antioxidant and antineoplastic effects^10,11^. Studies also show that it can suppress the inflammatory progression in human osteoarthritic chondrocytes^12^, and attenuate the arthritic symptoms in a collagen-induced mouse model of OA^13^. There is evidence suggesting that PD mediates these effects by modulating autophagy, and can significantly reduce apoptosis by increasing the autophagy flux^14,15^. Autophagy is highly conserved catabolic process involved in maintaining homeostasis within cells as well as recycling damaged cytoplasmic materials^16,17^, and is also involved in osteoarthritic progression^18^. It is tightly regulated by several pathways, including the MAPK, PI3K/Akt and AMPK signaling pathways^19^.

Based on these findings so far, we hypothesized that PD attenuates the progression of OA by regulating autophagy via the MAPK and PI3K/Akt signaling pathways. To verify our hypothesis, we established a rat model of OA by ACLT (anterior cruciate ligament resection) and simulated OA *in vitro* by treating primary chondrocytes with IL-1β, and subjected both models to PD treatment, and the association with the autophagy-related signaling pathways during the treatment period was provided by 3-methyladenine (3-MA), which can inhibit autophagy. We show for the first time that PD restores chondrocyte function by inducing autophagy, thus providing a novel therapeutic option for OA.

## Material and Methods

### Reagents

Polydatin (purity ≥ 95%), recombinant rat IL-1β, 3-MA, and type II collagenase came from Sigma (St Louis, MO, USA). The enzyme-linked immunosorbent assay (ELISA) kits for TNF-α and IL-6 were purchased from Cusabio (San Diego, CA, USA). Lentivirus expressing RFP-GFP–microtubule-associated protein light chain 3 (RFP-GFP–LC3) came from Genomeditech (Shanghai, China). The antibodies against GAPDH, Col I, Col II, TNF-α, IL-6, Akt, p-Akt, PI3K and p-PI3K were purchased from Abcam (Cambridge, MA, USA), those targeting LC3, mTOR, p-mTOR, ERK, p-ERK, JNK, p-JNK, P38 and p-P38 from Cell Signaling Technology (Beverly, MA, USA), and other antibodies targeting Beclin-1 from Novus Biologicals (Littleton, CO, USA). DyLight™ 800 4X PEG conjugated secondary antibody was from Cell Signaling Technology (Beverly, MA, USA).

RETRACTED

### Isolation of primary rat chondrocytes

Primary cartilage pieces were isolated from Sprague–Dawley (SD) rats (3–7 days old), minced, and dissociated with 2 mg/ml type II collagenase for 4 hours at 37 °C. Chondrocytes were harvested and re-suspended in α-MEM (Hyclone, Logan, UT, USA) containing 10% FBS (Hyclone) and 1% penicillin/streptomycin (Solarbio, Beijing, China). Cells were grown at 37 °C in a 5% CO_2_ humidified incubator. Cells were grown until 80%–90% confluent, and then passaged 1:3, and the passage 2 cells were used for further experiments. The animal protocol was approved by the Animal Ethical Committee of Animal Resources Centre of Guangxi Medical University (Nanning, Guangxi, China; ethic cord: 201805004). All methods for animal experiments were performed in accordance with relevant guidelines and regulations.

### Establishment of *in vitro* OA model and PD treatment

To determine the optimum concentration of PD for the chondrocytes, the cells were seeded in 96-well plates at the density of 5 × 10^3^ cells/well prior to treatment using PD (0.31–1280 μg/ml) alone, or with different PD doses (0.31–160 μg/ml) and 10 ng/ml IL-1β for 24 h. Viability was then assessed via adding 10 μl of 5 mg/ml MTT (3-(4,5-Dimethylthiazol-2-yl)-2,5-diphenyltetrazolium bromide) solution per well, and incubating at 37 °C for 4 h in the dark. After discarding this solution, 150 μl dimethyl sulfoxide (DMSO, Sigma-Aldrich) was added per well, and absorbance at 570 nm was assessed via Multiskan GO microplate reader (Thermo Fisher Scientific). The experiment was repeated in triplicates and based on the results, 10 μg/ml PD was selected for the subsequent experiments. The OA model was established by treating the chondrocytes with 10 ng/ml IL-1β, and cells were treated using PD with or without the autophagy inhibitor 3-MA (5 mM) for 24 h. Suitable untreated controls were also included. Cell proliferation and viability were determined by MTT assay as described.

### Cytological staining

The chondrocytes cultured in 24-well plates were followed by fixation for 30 min in 4% paraformaldehyde, and staining using hematoxylin and eosin (HE) (Solarbio, Bejing, China), toluidine blue (Boster, Wuhan, China) and safranin O (Solarbio) as per the instructions of the respective kits. The stained cells were dehydrated through an ethanol gradient, after which slides were sealed and assessed via microscope (Olympus, Japan).

RETRACTED

### Dual staining with fluorescein diacetate (FDA) and propidium iodide (PI)

Harvested chondrocytes were incubated with 2 µM FDA (Invitrogen Life Technologies, CA, USA) and 2 µg/L PI (Invitrogen) for 5 min at 37 °C in the dark. The live and dead cells were simultaneously evaluated via laser scanning confocal microscopy (Nikon A1, Japan).

### Annexin V and PI staining

The differentially-treated chondrocytes were harvested and re-suspended in Annexin V-FITC and PI working solution (Thermo Fisher Scientific), and incubated at 4 °C protected from light. A total of 1 × 10^4^ cells per sample were acquired by flow cytometry (BD Biosciences), and the percentage of apoptotic and live cells were assessed using FlowJo software (Tree Star Inc. Ashland, OR, USA).

### Immunostaining

Chondrocyte monolayers and cartilage sections were pretreated with 3% hydrogen peroxide, blocked with 10% normal goat serum (Gibco), and probed with primary antibodies against Col II (1:400), Col I (1:200), IL-6 (1:200) and TNF-α(1:200) overnight at 4 °C. After probing with the biotin-labeled IgG secondary antibody (1:200, ZhongShan Golden Bridge, Beijing, China), the samples were exposed to diaminobenzidine (DAB) (Boster, Wuhan, China) prior to hematoxylin counterstaining. Stained monolayers/sections were viewed via upright microscope (Olympus, Japan).

### Intracellular ROS measurement

Intracellular ROS was measured using a fluorescent 2,7-dichlorodihydro-fluorescein diacetate (DCFH-DA) probe kit (Nanjing Jiancheng Bioengineering Research Institute, Nanjing, China) based on provided directions. Briefly, the suitably treated chondrocytes were incubated with 10 μM DCFH‐DA at 37 °C for 30 min, after which flow cytometry was used to assess fluorescence, followed by FlowJo software analysis.

### Transmission electron microscopy (TEM)

The harvested chondrocytes were fixed for 24 h using 2.5% glutaraldehyde, after which 1% osmium tetroxide was used for 1 h at 4 °C for post-fixation. After staining with 2% uranyl acetate, the chondrocytes were dehydrated through an acetone gradient and embedded into araldite. Sample sections were cut and stained with toluidine blue, and observed by TEM (Hitachi, Tokyo, Japan).

### Measurement of autophagy flux

The stubRFP-sensGFP-LC3 lentivirus were constructed by Genechem Co (Shanghai, China). The primary passage 1 chondrocytes were seeded in 6-well plates, and after overnight culture were transduced with the lentivirus in serum-free medium at a multiplicity of infection (MOI) of 50. Complete α-MEM was used to replace media 12 h post infection, and the cells was grown for 24 h further while being treated with IL-1β, PD and 3-MA. The autophagic flux was observed using a laser scanning confocal microscope (Nikon America Inc., Melville, NY), and the stubRFP and sensGFP punctae were counted manually in at least 40 cells per sample.

RETRACTED

### Monodansylcadaverine (MDC) staining

The chondrocytes were stained using 0.05 mM MDC (Sigma, USA) to detect the autophagic vacuoles based on provided instructions, and cells were then assessed via laser scanning confocal microscopy as above.

### Establishment of *in vivo* OA model and treatment

Animal use in this study was approved by Animal care and use committee at Guangxi Medical University, Nanning, China. A total of 50 male Sprague-Dawley (SD) rats weighing 210−240 g were obtained from the Guangxi Medical University. The Guangxi Medical University Committee of Animal care and use approved all animal surgery procedures (protocol#: 201805005). The rats were anesthetized with 2% pentobarbital sodium solution via intraperitoneal injection, and ACLT was performed on the right hind limb to induce arthritis as previously described^20^. For the sham-operated controls, a similar incision was made on the left hind limb but the ligaments were left intact. The rats were allowed to recover for 4 weeks after surgery, and then given intra-articular injections of 0.2 ml PD (10 µg/ml) or PBS (OA group) once weekly for 4 or 8 weeks. All methods for animal experiments were performed in accordance with relevant guidelines and regulations.

### International cartilage repair society (ICRS) evaluation

The cartilage was harvested from the different animal groups, and macroscopically examined and graded according to the ICRS criteria^21^ by three independent observers blinded to the experimental conditions. The tissues were scored as: Grade 0 – normal, Grade 1 – soft indentation with superficial fissures and cracks, Grade 2 – lesions extending down to 50% of the cartilage depth, Grade 3 – cartilage defects extending to the calcified layer, and Grade 4 – severely deformed, with lesions extending through the subchondral bone.

### Histo-morphometric measurement

The harvested cartilages were fixed in 4% paraformaldehyde for 24 h, and decalcified in 0.5 M EDTA containing 8% hydrochloric acid for 3 to 4 weeks. The decalcified cartilages were embedded in paraffin and cut into 5 mm-thick sections, and stained with H&E, Saf-O/Fast Green and Masson dyes. The stained sections were observed using an upright microscope (OLYMPUS, Japan), and evaluated thrice and graded by 3 independent researchers using the Mankin histological criteria (Table 1)^22^.

**Table 1:** Mankin score (criteria for histological evaluation).

Item	Grade/classification	Grade
Structural intergrity	Normal	0
	Irregular Surface	1
	Pannus formation	2
	Fissures into transitional layer	3
	Fissures into emmiting layer	4
	Fissures into calcified layer	5
	Complete disorganization	6
Cells	Normal	0
	Hypercellularity	1
	Cloning	2
	Hypocellularity	3
Safranin-O staining	Normal	0
	Slight reduction	1
	Moderate reduction	2
	Severe reduction	3
	No dye noted	4
Tidemark intergrity	Normal	0
	Disruption	1

RETRACTED

### Enzyme-linked immunosorbent assay (ELISA)

Blood samples were coagulated at room temperature, and centrifuged at 3500 rpm for 15 min to separate the serum. The serum levels of TNF-α and IL-6 were quantified using the respective ELISA kits (Cusabio, San Diego, CA, USA) according to the manufacturer’s instructions.

### Total RNA isolation and quantitative RT-PCR (qRT-PCR)

Trizol reagent (Invitrogen) was used to isolate total chondrocyte RNA, followed by use of a RNeasy mini kit (QIAGEN, Valencia, CA, USA) for RNA purification. A total of 1 mg of total RNA per sample was reverse transcribed using a Transcriptor First- strand cDNA synthesis kit (Roche, Basel, Switzerland). SYBR Green master mix was used for qRT-PCR on an Applied Biosystems 7500 Real Time Cycler (Applied Biosystems, CA, USA). PCR conditions were as follows: 95 °C, 10 min, then 40 cycles of 95 °C, 15 sec and 60 °C, 1 min, followed by a standard melting curve. Sample was assessed in triplicates, with gene expression assessed based on the 2^−ΔΔCT^ method and GAPDH used for normalization. The primer pairs for target genes are listed in Table 2.

**Table 2:** Primer sequences used in qRT-PCR experiments.

Gene	Primer	Primer sequence (5′ to 3′)	Product size (bp)
GAPDH	Forward	AGTGCCAGCCTCGTCTCATA	77
	Reverse	GGTAACCAGGCGTCCGATAC	
Col II	Forward	ACGCTCAAGTCGCTGAACAACC	128
	Reverse	ATCCAGTAGTCTCCGCTCTTCCAC	
Col I	Forward	TGTTGGTCCTGCTGGCAAGAATG	145
	Reverse	GTCACCTTGTTCGCCTGTCTCAC	
ACAN	Forward	CTGATCCACTGTCCAAGCACCATG	131
	Reverse	ATCCACGCCAGGCTCCACTC	
SOX9	Forward	TCAACGGCTCCAGCAAGAACAAG	194
	Reverse	CTCCGCCTCCTCCACGAAGG	
MMP-13	Forward	AACCAAGATGTGGAGTGCCTGATG	167
	Reverse	CACATCAGACCAGACCTTGAAGGC	
IL-6	Forward	AGGAGTGGCTAAGGACCAAGACC	85
	Reverse	TGCCGAGTAGACCTCATAGTGACC	
TNF-α	Forward	GCATGATCCGAGATGTGGAACTGG	113
	Reverse	CGCCACGAGCAGGAATGAGAAG	
BAX	Forward	CCAGGACGCATCCACCAAGAAG	138
	Reverse	GCTGCCACACGGAAGAAGACC	
Bcl-2	Forward	ACGGTGGTGGAGGAACTCTTCAG	168
	Reverse	GGTGTGCAGATGCCGGTTCAG	
caspase-3	Forward	GTACAGAGCTGGACTGCGGTATTG	84
	Reverse	AGTCGGCCTCCACTGGTATCTTC	

GAPDH, glyceraldehyde-3-phosphate dehydrogenase; Col II, collagen type II; Col I, collagen type I; ACAN, aggrecan; SOX9, SRY box 9; MMP-13, matrix metallopeptidase-13; Il-6, interleukin-6; TNF-α, tumor necrosis factor-α; BAX, BCL2 associated X; Bcl-2, B cell leukemia-2.

RETRACTED

### Western blotting

RIPA Lysis Buffer (Beyotime, Beijing, China) containing phenylmethanesulfonyl fluoride (PMSF) (Beyotime, China) was used to extract protein from cartilage samples. Equal protein quantities 60 µg were denatured using SDS-PAGE loading buffer, separated through a 6% and 15% polyacrylamide gel and transferred onto a PVDF membrane (Millipore, Billerica, MA, USA). Primary antibodies against Col I, IL-6, TNF-α Beclin-1, LC3, mTOR, p-mTOR, Akt, p-Akt, PI3K, p-PI3K, ERK, p-ERK, JNK, p-JNK, P38, p-P38 (1:1000), and GAPDH (1:10000) were then used to probe blots at 4 °C overnight. Blots were washed thrice using PBST, after which they were probed using an appropriate DyLight™ 800 4X PEG conjugated secondary antibody (1:10000, Cell Signaling Technology) for 1 h. An Odyssey Infrared Imaging System was used to identify protein bands, and protein levels were quantified relative to the GAPDH loading control in the ImageJ software (NIH, Bethesda, Maryland, USA).

### Statistical analysis

Data were presented as mean ± SD, and assessed using SPSS17.0. Parametric data were compared via one way analysis of variance (ANOVA) with LSD (least significant difference) post-hoc tests, and non-parametric data was assessed via Mann-Whitney’s test. P values < 0.05 was the significance threshold.

## Results

### PD protects chondrocytes against IL-1β-induced apoptosis and structural disintegration

The chemical properties of PD are summarized in Fig. 1A. The chondrocytes were treated with varying concentrations of PD, and no apparent toxicity was seen for doses between 0.31 to 160 μg/ml (Fig. 1B), however, toxic was observed at high concentrations (≥320 μg/ml). In addition, IL-1β-treated chondrocytes exposed to 2.5, 5, 10, 20 and 40 μg/ml PD showed a significant increase in viability (Fig. 1C). Since optimal effects were seen with 10 μg/ml, it was selected for subsequent experiments.

**Figure 1:** Chondro-protective effects of PD on IL-1β-induced chondrocytes. (**A**) Chemical structures of PD. MTT assay was applied to detect the cytotoxicity of PD on chondrocytes with (**C**) or without (**B**) IL-1β. Values are the means ± SD (**p < 0.01, ***p < 0.001 indicate the significant difference amount the experiments, n = 5). After cultured with IL-1β, PD and 3-MA for 24 h, cell proliferation was determined by MTT assay (**D**). Values are the means ± SD (n = 5). Bars with different letters are significantly different from each other at *p* < 0.05 and those with the same letter exhibit no significant difference. Meanwhile, (**E**) H&E, (**F**) Saf-O and (**G**) FDA/PI staining of chondrocytes were applied for cell morphology, GAG production, and viability. Original magnification × 200 (scale bar, 300 μm).

RETRACTED

The typical round morphology of cultured chondrocytes (Fig. 1E) was affected by IL-1β, which also reduced the number of colonies. PD effectively rescued chondrocyte loss and resulted in the formation of cell clumps. In addition, PD treatment intensified safranin O staining (Fig. 1F), indicating increased secretion of glycosaminoglycan (GAG) chondroitin sulfate which was the structural component of cartilage. In addition, PD abrogated the inhibitory effects of IL-1β on cell proliferation and increased the proportion of viable cells (Fig. 1D,G). Interestingly, the autophagy inhibitor 3-MA reversed the protective effects of PD on chondrocyte proliferation, viability and structural integrity (Fig. 1D–G).

IL-1β also increased intracellular ROS levels, measured in terms of DCA fluorescence, to 34.67 ± 2.07. PD significantly reduced the production of ROS by 66.08%, and this effect was abrogated by 3-MA (Fig. 2A,B). Similarly, PD also reversed the up-regulation of the pro-apoptotic proteins BAX and caspase-3, and the down-regulation of the anti-apoptotic Bcl-2 in IL-1β-treated cells, and increased the Bcl-2/BAX ratio (Fig. 2C–F). In addition, the percentage of live chondrocytes was also significantly induced upon PD treatment (Fig. 2,H). Taken together, these results demonstrate that PD alleviates the pathological changes in chondrocytes by blocking intracellular ROS generation and apoptosis, and these effects are likely mediated via autophagy activation.

**Figure 2:** PD protects chondrocytes against IL-1β-induced apoptosis and ROS generation. *In vitro* pretreated with PD and 3-MA, representative ROS (**A**,**B**) and the percentage of live cells (**G**,**H**) was measured and quantitative counted by flow cytometry. (**C**–**F**) qRT-PCR was performed to analyze the apoptosis-related gene expression levels (Bcl-2, BAX, caspase-3, and the ratio of Bcl-2/BAX) *in vitro*. Bars with different letters are significantly different from each other at *p* < 0.05 and those with the same letter exhibit no significant difference. Values are the means ± SD (n = 5).

### PD restores chondrocyte function both *in vitro* and *in vivo*

Administration of PD effectively suppressed the IL-1β-induced increase in Col I and inflammatory factors like IL-6, TNF-α and MMP-13, and restored cartilage-specific markers including Col II, SOX9 and ACAN in the chondrocytes (Fig. 3A–L). Predictably, the inhibition of autophagy by 3-MA abrogated the restorative effects of PD *in vitro*. Consistent with the *in vitro* findings, the cartilage of the untreated OA-modeled rats harbored only a few Col II-positive chondrocytes in the superficial layers (Fig. 4H), which increased significantly following 4 or 8-weeks of PD treatment. In addition, the Col II and ACAN mRNA levels were significantly increased in the cartilages of PD-treated compared to the untreated OA rats (Fig. 4K,L), whereas the *in situ* levels of IL-6 and TNF-α were both significantly lower after PD treatment (Fig. 4I,J,M,N). Taken together, PD reverses cartilage destruction accompanying OA by blocking inflammatory progression, promoting cartilage matrix repair, and inhibiting de-differentiation of chondrocytes.

RETRACTED

**Figure 3:** PD restores chondrocyte function *in vitro*. (**A**–**D**) Western blot of Col I, IL-6, and TNF-α in different groups were detected respectively and the semi-quantitative analysis of Col I/GAPDH, IL-6/GAPDH, and TNF-α/GAPDH are shown. (**E**–**K**) qRT-PCR was performed to determine the expression levels of (**E**–**H**) Col I, Col II, SOX9 and ACAN and (**I**–**K**) osteoarthritis relative gene (IL-6, TNF-α and MMP-13). Values are the means ± SD, n = 5. Bars with different letters are significantly different from each other at *p* < 0.05 and those with the same letter exhibit no significant difference. (**L**) Immunohistochemical staining images revealed the presence of Col I, Col II, IL-6, and TNF-α. Original magnification × 200 (scale bar, 300 μm).

**Figure 4:** Protection effects of PD on the treatment of OA. *In vivo* cartilage repair at 4 and 8 weeks post-surgery, (**A**) Macroscopic appearance and (**B**) ICRS scores of femoral condyles from OA rat were detected. (**C**–**E**) H&E staining, Saf-O/Fast Green staining, and Masson staining were performed in sections of cartilage. Original magnification × 40 (scale bar, 2,000 μm). (**F**,**G**) Histological score of articular cartilage was determined. (**H**–**J**) Immunohistochemical staining of Col II, IL-6, and TNF-α was performed in sections of cartilage. Original magnification × 80 and × 320. (**K**–**N**) qRT-PCR was performed to analyze the expression of Col II, ACAN, TNF-α, and IL-6 genes in cartilage at 4 and 8 weeks. Meanwhile, serum levels of (**O**) IL-6, and (**P**) TNF-α were determined using ELISA kits. Values are the means ± SD (n = 10). Bars with different letters are significantly different from each other at *p* < 0.05 and those with the same letter exhibit no significant difference.

### PD activates the autophagic flux in chondrocytes

As shown in Fig. 5H, PD significantly increased the number of MDC-labeled autophagic vacuoles in the IL-1β-stimulated chondrocytes, along with Beclin-1 levels and the LC3-II/LC3-I ratio (Fig. 5D–F), all indicative of autophagy. In addition, PD treatment decreased the ratio of p-mTOR/mTOR compared to that in the IL-1β group (Fig. 5G). Upregulation of autophagy markers and the presence of numerous autophagic vaculoes however are static indicators of autophagy. To observe the autophagic flux, therefore, we transduced RFP-GFP–LC3 into chondrocytes to simultaneously track the autophagosomes (yellow punctae that are a combination of red and green fluorescence) and autophagolysosomes (red punctae). PD treatment significantly increased the proportion of autophagolysosomes in the cytoplasm of IL-1β-treated chondrocytes (Fig. 5B,C), indicating autophagy induction. Finally, transmission electron microscopy (TEM) validated the increased number of autophagosomes, autophagic vesicles and autolysosomes in the PD-treated chondrocytes (Fig. 5A). As expected, 3-MA partially inhibited the autophagy inducing effects of PD. Taken together, PD activates the autophagic flux in the IL-1β-treated chondrocytes which, based on the results so far, is the underlying basis of its regenerative effects.

RETRACTED

**Figure 5:** Effects of PD on autophagic flux in cultured chondrocytes *in vitro*. (**A**) TEM images of the autophaghic change in chondrocytes. Single arrow: autophagolysosome and autophagosome with double membrane structure. Original magnification × 30000 (scale bar, 500 nm). (**B**) Cells transfected with adenovirus harbouring tandem fluorescent mRFP-GFP-LC3 for 24 h were subjected to different treatments. Representative pictures of immunofluorescent chondrocytes expressing mRFP-GFP-LC3. GFP dots are green, and mRFP dots are red. Original magnification × 1600 (scale bar, 20 μm). (**C**) Semi-quantitative analysis of autophagosomes (AP; yellow dots in merged images) and autolysosomes (AL; red only dots in merged images). (**D**) Western blot of LC3, Beclin1, and mTOR in different groups were detected respectively and the semi-quantitative analysis of LC3 II/I ratio, Beclin1/GAPDH, and mTOR/GAPDH are shown. (**H**) Representative pictures of MDC staining. Original magnification × 1600 (scale bar, 20 μm). Values are the means ± SD (n = 5). Bars with different letters are significantly different from each other at *p* < 0.05 and those with the same letter exhibit no significant difference.

### PD regenerates the cartilage *in vivo* by promoting chondrogenesis and blocking inflammation

Macroscopic examination of the femoral distal heads of the untreated OA rats showed thick, hard and yellowish fibrotic tissue, ossification and reduced articular cartilage thickness over the entire knee joint surface. Administration of PD markedly reduced fibrosis, and resulted in a more uniform appearance and the formation of soft neo-cartilage (Fig. 4A). The ICRS scores decreased significantly in the PD-treated group by 1.9 ± 0.2 and 1.5 ± 0.5 folds at 4 and 8 weeks respectively, compared to the untreated OA rats (Fig. 4B). Furthermore, knee cartilage sections of the untreated OA animals showed pale Saf-O staining, which deepened in the PD group rats (Fig. 4D) indicating progressively increasing proteoglycan synthesis and chondrogenesis. HE and Masson staining showed fewer and sporadically distributed chondrocytes, reduced thickness and extensive fibrosis in the cartilage of untreated OA rats (Fig. 4C,E). Treatment with PD significantly ameliorated the cartilage damage, and decreased the infiltration of inflammatory cells and fissure formation. Cartilage repair wa**s** quantified in terms of the modified Mankin score, which was lowest in the PD group after 4 and 8 weeks of therapy compared to the untreated OA group (Fig. 4F,G). In addition, the post-ACLT serum levels of TNF-α and IL-6 were markedly reduced, and the downregulation of TNF-α to baseline levels by PD (Fig. 4O,P). Taken together, PD effectively repairs the cartilage damage following ACLT by promoting neo-chondrogenesis, and inhibiting the inflammatory response.

RETRACTED

### PD ameliorates autophagy development by modulating the MAPK and PI3K/Akt signaling pathways

To further elucidate the potential mechanism underlying PD-induced autophagy in the injured chondrocytes, we analyzed the levels of the mediators of MAPK and PI3K/Akt pathways in the differentially-treated cells. As shown in Fig. 6A, IL-1β increased the levels of phosphorylated JNK, P38, ERK, PI3K and Akt, which was diminished by PD in a concentration-dependent manner. At the dose of 10 μg/ml, the ratio of above markers were restored largest. These findings indicate that inhibition of MAPK and PI3K/Akt signaling, which are the key upstream suppressors of mTOR, is the possible mechanism by which PD restores autophagy. In the *in vivo* OA model as well, PD significantly down-regulated the p-P38/P38, p-ERK/ERK, p-JNK/JNK, p-PI3K/PI3K, and p-Akt/Akt ratios (Fig. 6B). A scheme of signaling pathways involved in the anti-osteoarthritic effects of PD is presented in Fig. 7.

**Figure 6:** *In vitro* and *in vivo* signaling pathway research. After pre-cultured with different concentrations (2.5, 5, and 10 μg/ml) of PD for 24 h *in vitro* (**A**), and treated with 10 μg/ml of PD for 8 W *in vivo* (**B**), Western Blot was used to analyze the progression of the expression of MAPK and PI3K/AKT signaling pathway proteins p-Akt, Akt, p-PI3K, PI3K, p-JNK, JNK, p-P38, P38, p-ERK, and ERK. Bars with different letters are significantly different from each other at *p* < 0.05 and those with the same letter exhibit no significant difference. Values are the means ± SD (n = 5).

RETRACTED

**Figure 7:** Schematic description of relative signaling pathways that activated by PD. ( → Direct Stimulatory Modification, ┤Direct Inhibitory Modification).

## Discussion

Polydatin is a plant-derived anti-inflammatory and antioxidant compound that is known to repress pro-inflammatory chemokine secretion in arthritis^13^, as well in cultured human OA chondrocytes^12^. Consistent with this, we found that PD enhanced chondrocyte viability and proliferation (Fig. 1D,G), increased deposition of chondroitin sulfate (Fig. 1F), and restored the pebble-like morphology of chondrocytes (Fig. 1E) stimulated by the pro-inflammatory IL-1β. In addition, PD treatment also restored chondrocyte markers expression of Col II, SOX9 and ACAN, and downregulated the de-differentiation marker Col I (Fig. 3A,B,E–H,L). The pro-inflammatory cytokines IL-6 and TNF-α^23^, and the ECM proteinase MMP-13^24^, were also reduced *in vitro* following PD treatment (Fig. 3A,C,D,I–L). Consistent with the *in vitro* findings, administration of PD in the ACLT-induced OA model alleviated cartilaginous damage, as indicated by the normalization of ICRS scores (Fig. 4A,B), increased collagen deposition (Fig. 4D,E) and greater structural uniformity (Fig. 4C,G). In addition, PD also increased Col II and ACAN expression in the cartilage (Fig. 4H,K,L) and decreased the serum levels of IL-6 and TNF-α(Fig. 4O,P).

The generation of intracellular ROS is a major pathological driver of apoptosis in the chondrocytes^25^, which in turn plays a vital role in triggering inflammation^26,27^. IL-1β stimulation significantly increased ROS levels in the chondrocytes (Fig. 2A,B), decreased cellular proliferation (Fig. 1D) and induced apoptosis, as indicated by the up-regulation of BAX and caspase-3 and suppression of the anti-apoptotic Bcl-2 (Fig. 2C–F). PD treatment not only reversed the expression pattern of the apoptosis-related factors and increased the percentage of live cells (Fig. 2G,H), but also inhibited ROS generation. An increase in oxidative stress predisposes chondrocytes to a dysfunctional antioxidant response and apoptosis^28^. Therefore, we can surmise that PD inhibits apoptosis in the injured chondrocytes by attenuating oxidative stress, and that ROS could be a potential therapeutic target in OA.

Autophagy is a catabolic process wherein damaged proteins and organelles are phagocytosed and degraded to maintain energy levels and support organelle renewal^29^. It is often activated during stress conditions like hypoxia, starvation and accumulation of ROS, in order to prevent apoptosis and maintain cellular homeostasis^30–32^. However, an unfavorable microenvironment, such as that of the arthritic cartilage, can suppress autophagy^33^. Indeed, we found that LC3-II/LC3-I and Beclin-1 levels were significantly suppressed in the IL-1β-induced chondrocytes, and restored upon PD treatment (Fig. 5D–G). In addition, PD also increased the autophagic flux and increased autolysosomes generation in the IL-1β-treated chondrocytes (Fig. 5A–C). Consistent with this, the PD-treated OA chondrocytes showed significantly lower levels of ROS and inflammatory factors. The phosphoinositide 3-kinase (PI3K) blocker 3-MA is routinely used as an inhibitor of autophagy^34^, and markedly abrogated the effects of PD on apoptosis and ROS generation. The expression levels of inflammation cytokines (IL-6, TNF- α, and MMP-13) and de-differentiation markers (Col I) were also significantly increased by treatment with 3-MA, this result is consistent with the findings of autophagy protection in existing researches^35–37^, one possible explanation is that induction of autophagy plays the key role in maintaining the phenotype of chondrocyte and inhibiting inflammatory response. In short, our findings reveal that PD likely relieves symptoms by activating autophagy, however, more studies are required to clarify the further mechanism.

RETRACTED

Mammalian target of rapamycin (mTOR) plays a key role in suppressing autophagy, and is regulated by multiple upstream signaling pathways, including the MAPK and PI3K/Akt pathways^38,39^. The MAPK pathway is also a key pro-inflammatory pathway that has been linked to the pathogenesis of OA^40^. In our study, PD significantly downregulated the phosphorylated MAPKs as well as mTOR in the chondrocytes in a concentration-dependent manner (Figs 5G and 6A,B), thereby supporting the modulatory role of PD on the mTOR signaling pathway^14^. The PI3K/AKT pathway also is important for controlling the apoptosis and inflammatory activity in chondrocytes. Following PI3K activation, the downstream AKT is phosphorylated, thereby affecting BAX, Bcl-2 and caspase-3 expression and influencing apoptosis^41^. In this study, PD impaired PI3K, AKT and mTOR phosphorylation (Fig. 6A,B), with mTOR being a downstream target of AKT as well^42^. Specifically, some studies reveal that the inhibition effect of polydatin on mTOR is related to the endoplasmic reticulum (ER) stress and glucose metabolism pathway^43,44^. Indeed, ER stress, glucose metabolism, MAPK, and PI3K can modulate autophagy via regulating mTOR, however, their interactions during the polydatin treatment are still unclear. Taken together, administration of PD inhibited inflammatory progression in the arthritic cartilage that was at least partly mediated by the suppression of MAPK and PI3K/AKT cascades, leading to mTOR inhibition.

RETRACTED

In conclusion, PD partially inhibits IL-1β-triggered inflammation and ACLT in chondrocytes. The chondro-protective effects of PD were associated with apoptosis inhibition, reduced ROS production and autophagy activation, and mediated via a repressed MAPK and PI3K/AKT/mTOR axis. Although our findings are preliminary, they provide a novel anti-OA therapeutic strategy which needs to be validated further by clinical studies.

## Data Availability

The data used to support the findings of this study are available from the corresponding author upon request.
